This article has been retracted.

# Effect of Medical Image Fusion in the Treatment of Poststroke Limb Dysfunction with Acupuncture and Moxibustion of Traditional Chinese Medicine

**DOI:** 10.1155/2022/8380251

**Published:** 2022-09-29

**Authors:** Aiping Feng, Wanliang Guo, Yong Jia

**Affiliations:** Zhangye Second People's Hospital, Zhangye, 734000 Gansu, China

## Abstract

According to relevant data, the morbidity and mortality of strokes in China remain high. Without effective treatment, stroke morbidity and mortality will continue to rise, which may become the second leading disease in the world. With the nonstop advancement and improvement of clinical innovation in China, the death pace of stroke patients has dropped altogether. After clinical treatment, the patient actually showed a progression of sequelae, which made it challenging to work on the personal satisfaction of the patient. The purpose for this paper was to concentrate on the impact of medical image fusion in the treatment of poststroke appendage brokenness with TCM needle therapy. The related concepts of medical image fusion and the meaning of acupuncture and moxibustion in traditional Chinese medicine, stroke, and limb dysfunction were introduced. In this study, acupuncture and moxibustion were analyzed to explore the therapeutic effect of this type of therapy on upper extremity dysfunction caused by phlegm and blood stasis blocking collaterals and to provide a scientific method for the treatment and efficacy judgment of upper extremity motor dysfunction after stroke. Before the treatment measures were taken, there was no significant difference in the general data and all index scores between the two groups (*P* > 0.05), and there was no significant difference in the baseline data, reflecting high balance and comparability. In the following 3 months of treatment, the FMA score, NIHSS score, BI list, and VAS score of the two groups of patients were essentially not quite the same as those before treatment (*P* < 0.05). When treatment, there was a huge contrast between the trial group and the control group (*P* < 0.05). The finish of the trial in this paper is that needle therapy joined with pricking and measuring can essentially work on the engine capability of stroke patients with furthest point brokenness brought about by mucus and blood balance impeding securities.

## 1. Introduction

Limb dysfunction is the biggest factor leading to disability in stroke patients, and restoring their limb function is an important task in treatment. The recovery of limb dysfunction after stroke basically goes through three stages: soft paralysis, hard paralysis, and recovery. The flaccid stage is mainly manifested as decreased or even disappearance of muscle strength, muscle tension, and inability of limbs to move voluntarily. Long-term atrophy and waste are caused by this, which affects the recovery of limb function, burdens the patient with heavy psychological pressure, and brings a heavy economic burden to the patient's family. Therefore, the flaccid period is a critical period for the recovery of limb dysfunction, and it is necessary to receive regular Chinese and Western medicine rehabilitation treatment as soon as possible.

Acupuncture and moxibustion in traditional Chinese medicine are important parts of traditional Chinese medicine with a history of five thousand years. Because of its unique characteristics and advantages, it has become the representative of traditional Chinese medicine culture. With the development of science and technology and social economy and the continuous improvement of people's living standards, the discipline of traditional Chinese medicine and acupuncture has also entered a period of rapid development. Computer technology has been widely studied and applied in clinical, teaching, and scientific research in the field of traditional Chinese medicine acupuncture and moxibustion. Medical image processing is one of the important technical means for diagnosing, treating, and diagnosing diseases by analyzing the multidimensional structure and function of tumors. It can not only display the anatomical details of the focal area but also display the blood flow, which improves the utilization of image information. The innovation of this paper is to further expand the scope of application of acupuncture and moxibustion in traditional Chinese medicine. At the same time, it provides a good theoretical basis for the diagnosis and treatment of upper limb dysfunction in patients after stroke. In addition, drug therapy is being explored for the treatment of the disease for which the desired effect is difficult to achieve.

## 2. Related Work

With the development of Chinese medicine, more and more scholars have conducted research on TCM acupuncture techniques. Chen et al.'s survey of Chinese acupuncture and moxibustion among foreigners in Shanghai reflected the international awareness, advantages and disadvantages, and overseas spread of Chinese acupuncture and moxibustion [1]. Liu et al. reviewed the development background of acupuncture instruments, the difficulties encountered in the development process, and the countermeasures and summarized the experience of standard formulation, aiming to provide methods and references for the development of acupuncture instruments in the future [2]. Si mainly reviewed the selection of acupoints, the location and depth of acupuncture, and other treatments recorded in published reports on the treatment of perimenopausal insomnia, hoping to be helpful to clinical treatment [3]. Anastasi et al. described the development of an acupuncture regimen used in a randomized controlled trial of diarrhea-predominant irritable bowel syndrome in adults [4]. However, the shortcoming of these studies is that the models constructed are not scientific enough.

With the improvement of social economy, medical image fusion technology has continuously started to prosper. Yin proposed a 3D image fusion strategy in view of tensor meager portrayal (TSR) [5]. Jarholiya performed two-level DWT decomposition on the image and then used an improved DC coefficient scaling method in the compressed DCT domain to enhance the contrast difference of multimodal images [6]. Tian et al. joined convolutional sparsity and heartbeat coupled brain organizations to propose a perceptual medical image fusion structure in light of morphological part examination [7]. Rani and Lalithakumari proposed a scale expansion model based clinical 2D image fusion technique, called 2D Double Density Wavelet Transform (2D-DDWT), which was utilized for the combination of human mind CT and MRI images [8]. The disadvantage of these examinations, in any case, is that the contemplations are not adequately extensive to adjust to additional perplexing circumstances.

## 3. Related Methods of Medical Image Fusion

### 3.1. Concept and Application of Image Fusion

#### 3.1.1. Concept of Image Fusion

Image fusion is an algorithm that fuses image data together to form a new image. Its main idea is to use a certain algorithm to fuse multiple imaging information of the same scene from image sensors working in different wavelength ranges and with different imaging mechanisms into a new image. Therefore, the fused image has higher reliability, less blur, better understandability, and is more suitable for human vision and computer detection, classification, recognition, understanding, and other processing. It alludes to images of similar objective or pictures gathered from numerous directs at various times in similar channel or pictures of a similar objective gathered at various times in a similar channel. Through certain image processing, information is extracted from each channel, and finally, the image is fused into an observation image or further processed [9, 10].

#### 3.1.2. Advantages of Image Fusion

(1) Data redundancy can be reduced. (2) Image fusion processing can learn from each other. (3) By using multisensors for multisource fusion analysis, the characteristics of each image can be better utilized, and different image information can be properly fused to provide more comprehensive information.

#### 3.1.3. General Model and Steps of Image Fusion

The general model of image fusion is shown in Figure 1 [11].

Among them, spatial registration is an important part of image fusion. Usually, the registration method is selected by itself according to the difference of the images collected by different sensors. The fusion method experiment in this paper is based on the registered image data, focusing on exploring information fusion technology and related algorithms. The steps of multisensor image fusion are as follows: the first step is to perform spatial registration of images collected by different sensors; the second step is to perform fusion operations on the registered images; the third step is to analyze and understand the fusion result images.

#### 3.1.4. Classification and Methods of Medical Image Fusion

There are different orders of medical image fusion technology, classified by imaging equipment, classified by fusion object, classified by image type, classified by image dimension, and classified by processing method. For clinical images, images of various modes have various qualities, and the necessities for medical image fusion are likewise exceptionally high, so image fusion is a truly challenging errand [12, 13]. Image fusion can be separated into three levels: pixel-level (crude information) fusion, highlight-level (or target-level) fusion, and choice-level fusion. The various leveled designs of image fusion are displayed in Figure 2.

Lately, with the extending of image fusion research, three image fusion technologies have been proposed: pixel-level image fusion, include-level image fusion, and choice-level image fusion [14].

Pixel-level image fusion can be isolated into two classes: spatial area and change space. Algorithms based on the spatial domain are easy to implement but have low computational complexity and poor accuracy. The main fusion process of transform domain image fusion is to first convert the source image to the transform domain and then use some fusion rules to process and inversely transform the reconstructed image. The advantage of pixel-level image fusion is that it can extract more detailed information of the source image, with high precision, which is convenient for researchers or machines to perform subsequent analysis and understanding of the image. Of course, the disadvantage is that all source images must be accurately registered before the fusion operation, and the fusion process takes a long time, resulting in poor real-time performance. And there are certain requirements for the instruments and equipment used for fusion. This degree of combination framework structure is displayed in Figure 3.

The main processing flow of feature-level image fusion is usually to first extract the required features in the images to be fused. The extracted features are then processed using a fusion method to obtain a fused image that preserves the features required for analysis to the greatest extent possible. At the same time, it effectively compresses the information, reduces the calculation amount of fusion processing, and realizes the real-time processing of image fusion. But its disadvantage is that it is easy to lose more useful source image data in the fusion process, so the information utilization rate of the source image is not high. The system architecture of feature-level image fusion is shown in Figure 4.

The main process of decision level fusion is to extract the target needed in the source image after preprocessing the source image. Then, the acquired targets are identified, and decisions are made for each target, respectively. According to certain criteria and the credibility of each decision, all decisions are processed accordingly, and finally, a global optimal joint decision is formed [15, 16]. The hierarchical fusion has the advantages of low amount of communication data, strong adaptability, and robustness. Because the decision-level image fusion is the final joint decision formed according to the preliminary decision conclusion, the information loss to the source image is also the largest. The level of fusion system architecture is shown in Figure 5.

The three level image fusion structures described above are closely related to each other, and the image fusion results of the lower level become the input of the higher level image fusion [17]. Considering the specific characteristics of medical images and many advantages of pixel-level image fusion, the medical image fusion algorithms used in the subsequent chapters of this paper are pixel-level image fusion methods.

### 3.2. Quality Evaluation of Fusion Images

The main purpose of medical image fusion is to obtain a comprehensive information including the lesion area and to maximize the preservation of important details such as the texture edge of the source image. And medical images with good human visual effects provide comprehensive and accurate information support for subsequent doctors to accurately diagnose the disease and formulate more reasonable treatment plans. Therefore, objective, accurate, and reasonable fusion image quality evaluation criteria are very critical.

#### 3.2.1. Subjective Evaluation Method

As the name implies, the subjective evaluation method means that researchers directly observe the image to be evaluated with their eyes and evaluate the image quality based on their subjective judgment [18]. Subjective evaluation methods are affected by external factors, such as whether the observer has relevant professional background knowledge, systematic training, and psychological and emotional stability. Therefore, the image evaluation results obtained by using subjective evaluation methods often vary from person to person. Subjective evaluation method is intuitive and easy to implement, but it is inefficient and requires a lot of human resources when evaluating a large number of images. Therefore, at present, subjective evaluation methods can only be used as qualitative analysis and reference for objective evaluation methods. The five-grade quality scale and obstruction scale of international general image subjective evaluation are shown in Table 1.

#### 3.2.2. Objective Evaluation Methods

Objective evaluation indexes are mainly defined according to some physical meanings of images, such as information state, gradient, and frequency. Objective evaluation indicators have the advantages of objective universality and high efficiency [19]. The objective evaluation methods at this stage are mainly divided into three categories according to the difference of the measurement targets: the evaluation index of the characteristics of the fusion image itself, the evaluation index of the relationship between the fusion image and the standard reference image, and the evaluation index of the relationship between the fusion image and the source image. *G* represents fusion image, *A* and *B* are source image, and *R* represents standard reference image.

*(1) Evaluation Indexes of Fusion Image Characteristics*.

- Information office

Information integrity is an objective evaluation index to quantify how much information an image contains. When the noise in the image is ignored, the high information integrity indicates that the image contains a large amount of data and rich useful information. The definition formula of information state is as follows:

(1) $$\begin{array}{c} E=\overset{W-1}{\underset{i=0}{\sum }}h_{i}\log_{2}h_{i}. \end{array}$$

In the formula, *h*_*i*_ is the ratio of the total number of all pixel points with gray value of *I* in the image to be tested to pixel points contained in the image, *i* = [0, 1, ⋯, *W* − 1], and *W* is the gray level of the image to be tested.

(b) Mean gradient

According to the definition, average gradient reveals the mutation degree of gray values between adjacent pixels of the whole image [20]. The larger the value is, the more details in the image and the clearer the fusion image will be. The definition formula is as follows:

(2) $$\begin{array}{c} AG=\frac{1}{U\times V}\overset{U}{\underset{x=1}{\sum }}\overset{V}{\underset{y=1}{\sum }}\sqrt{\frac{\Delta G_{x}^{2}+\Delta G_{y}^{2}}{2}}. \end{array}$$

In the above formula, Δ*G*_*x*_, Δ*G*_*y*_, respectively, represents the first-order difference between the gray values of pixel points at (*x*, *y*) and adjacent pixel points along the horizontal and vertical directions. *U* and *V* represent the matrix of *U* × *V* of the image to be tested.

(c) Standard deviation

The definition of standard deviation reflects the difference between the gray values of all pixels in the image and the mean value of the image. In the case of ignoring noise interference, it can be considered that the larger the standard deviation is, the more discrete the gray value in the image is, and the richer the detailed information such as texture edge is. The specific definition formula is as follows:

(3) $$\begin{array}{c} \sigma =\sqrt{\frac{\sum_{i=1}^{U}\sum_{j=1}^{V}{\left[g\left(i,j\right)-\mu \right]}^{2}}{U\times V}}. \end{array}$$

Among them, *μ* represents the mean value of the image, *U*, *V* represents the matrix of *U* row and *V* column of the image to be tested, and *g*(*i*, *j*) represents the gray value at the image (*I*., *j*).

(d) Spatial recurrence

Spatial recurrence is utilized to quantify the general movement of all pixels in the image in the even and vertical bearings [21, 22]. The particular definition formula is as the following:

(4) $$\begin{array}{c} \text{RF}=\sqrt{\frac{1}{U\times V}\overset{U}{\underset{i=1}{\sum }}\overset{V}{\underset{j=2}{\sum }}{\left[g\left(i,j\right)-g\left(i,j-1\right)\right]}^{2}},\\ \text{CF}=\sqrt{\frac{1}{U\times V}\overset{U}{\underset{i=2}{\sum }}\overset{V}{\underset{j=1}{\sum }}{\left[g\left(i,j\right)-g\left(i-1,j\right)\right]}^{2}},\\ \text{SF}=\sqrt{{\text{RF}}^{2}+{\text{CF}}^{2}}. \end{array}$$

In the above formulas, CF and RF are row and column frequencies, and SF is the overall spatial frequency of the image.

(e) Edge intensity

The edge intensity is used to measure the degree of grayscale change between the edge and its adjacent pixels in the image. This parameter reveals the richness of details such as edge texture in the fused image. Its definition formula is as follows:

(5) $$\begin{array}{c} EI=\left|\mathrm{grad}\left(g\left(x,y\right)\right)=\left|\nabla_{x}g\right|+\left|\nabla_{y}g\right|\right|. \end{array}$$

In the above formula, *g*(*x*, *y*) is the gray value, and ∇_*x*_*g* and ∇_*y*_*g* are the gradient values in the horizontal and vertical directions, respectively.

*(2) Evaluation Record of the Connection between the Fused Image and the Standard Reference Image*. This kind of assessment list essentially mirrors the distinction between the image to be tried and the standard image, and the standard image is required as a source of perspective to finish. The standard reference image is the image fusion of the best impact.

- Signal-to-commotion proportion

The signal-to-commotion proportion is principally used to work out the mathematical worth of the distinction between the image fusion and the standard reference image contrasted with the standard image, which mirrors the devotion of the image fusion. The particular recipe is as follows:

(6) $$\begin{array}{c} SNG=10\mathrm{lg}\frac{\sum_{i=1}^{U}\sum_{j=1}^{V}G{\left(i,j\right)}^{2}}{\sum_{i=1}^{U}\sum_{j=1}^{V}{\left[G\left(i,j\right)-R\left(i,j\right)\right]}^{2}}. \end{array}$$

Among them, *G*(*i*, *j*) and *R*(*i*, *j*) are *G* and *R* images.

(b) Correlation coefficient

The correlation coefficient is primarily used to gauge the relationship between the test picture and the standard picture. The more associated the intertwined picture is with the standard reference picture, the nearer the worth of Corr is to 1. The particular definition recipe is as the following:

(7) $$\begin{array}{c} \text{Corr}=\frac{\sum_{i=1}^{U}\sum_{j=1}^{V}\left|G\left(i,j\right)-\mu_{G}\right|\times \left|R\left(i,j\right)-\mu_{R}\right|}{\sqrt{\sum_{i=1}^{U}\sum_{j=1}^{V}{\left|G\left(i,j\right)-\mu_{G}\right|}^{2}\times {\left|R\left(i,j\right)-\mu_{R}\right|}^{2}}}. \end{array}$$

Among them, *G*(*i*, *j*) and *R*(*i*, *j*) represent *G* and *R* images, respectively, and *μ*_*G*_ and *μ*_*R*_ are the mean values of *G* and *R*.

(c) Degree of distortion

The level of twisting is utilized to quantify how much contortion of the *G* comparative with the *R* picture, and the more modest the worth, the better the nature of the picture to be tried. The particular definition formula is as the following:

(8) $$\begin{array}{c} DD=\frac{1}{U\times V}\overset{U}{\underset{i=1}{\sum }}\overset{V}{\underset{j=1}{\sum }}\left|G\left(i,j\right)-R\left(i,j\right)\right|. \end{array}$$

*(3) Evaluation Index of the Relationship between the Fusion Image and the Source Image*.

- Cross entropy

Cross entropy represents the degree of difference in the distribution of gray values between *G* and *A* and *B*. The larger the value, the less data *G* extracts from *A* and *B*. The specific definition formula is as follows:

(9) $$\begin{array}{c} Q=\overset{W-1}{\underset{i=0}{\sum }}h_{i}\log_{2}\frac{h_{i}}{s_{i}}. \end{array}$$

In the formula,

(10) $$\begin{array}{c} h_{i}=\left\{h_{0},h_{1},\cdots ,h_{i},\cdots ,h_{W-1}\right\},\\ s_{i}=\left\{s_{0},s_{1},\cdots ,s_{i},\cdots ,s_{W-1}\right\}. \end{array}$$

In practical applications, in order to comprehensively reflect the overall difference between the fused image and the source image, the average cross entropy is usually used to represent the following:

(11) $$\begin{array}{c} {\bar{Q}}_{GAB}=\frac{Q_{GA}+Q_{GB}}{2}. \end{array}$$

In the formula, *Q*_*GA*_ and *Q*_*GB*_ represent the cross-entropy of *G* with *A* and *B*, respectively.

(b) Amount of interactive information

The amount of interactive information is an important indicator that reflects how much information the fused image extracts from the source image. At the same time, it also reflects the similarity of the information distribution of the two images. MI_*GA*_ and MI_*GB*_ are the interactive information amounts of images *A*, *B*, and *G*, respectively, and the calculation formula is as follows:

(12) $$\begin{array}{c} {\text{MI}}_{GA}=\overset{W-1}{\underset{k=0}{\sum }}\overset{W-1}{\underset{i=0}{\sum }}h_{GA}\left(k,i\right)\log_{2}\frac{h_{GA}\left(k,i\right)}{h_{G}\left(k\right)h_{A}\left(i\right)},\\ {\text{MI}}_{GB}=\overset{W-1}{\underset{k=0}{\sum }}\overset{W-1}{\underset{i=0}{\sum }}h_{GB}\left(k,i\right)\log_{2}\frac{h_{GB}\left(k,i\right)}{h_{G}\left(k\right)h_{B}\left(i\right)}. \end{array}$$

The above formulas are the joint grayscale distribution of the two sets of images, respectively. In order to comprehensively calculate the amount of interactive information between *G* and *A* and *B*, usually the sum of MI_*GA*_ and MI_*GB*_ is directly taken as MI_*G*_^*AB*^, and the calculation formula is as follows:

(13) $$\begin{array}{c} {\text{MI}}_{G}^{AB}={\text{MI}}_{GA}+{\text{MI}}_{GB}. \end{array}$$

### 3.3. Understanding of Traditional Chinese Medicine on Stroke and Limb Dysfunction during Stroke Flaccid Paralysis

#### 3.3.1. Concept of Stroke

Stroke is known as the three major “killers” that seriously endanger human health together with heart disease and cancer. It is described by high dreariness, high mortality, high handicap rate, and high repeat rate. The 2015 China Stroke Prevention and Control Report stated that there are about 2 million new strokes every year, and the rapid growth rate is high every year, which is much higher than the average incidence of stroke in the world, and pointed out that stroke is the leading cause of death among Chinese residents. In recent years, the number of deaths due to stroke has decreased significantly due to residents' emphasis on stroke prevention and the improvement of medical staff's diagnosis and treatment level. However, the increase in the number of surviving stroke-disabled patients has led to an unabated increase in the stroke-disability rate in China.

#### 3.3.2. Understanding of TCM on Limb Dysfunction during Stroke Flaccid Paralysis

Limb dysfunction during stroke flaccid paralysis is mainly manifested as limb weakness and inability to move after stroke. In traditional Chinese medicine, there is no such name as “limb dysfunction during stroke flaccid paralysis.” According to its clinical manifestations, it can be classified into the categories of “slightly dry,”, “partially windy,” “partially useless,” etc., and some people classify it as “withering syndrome.” In “Lingshu • Fever”: “The symptoms of prickly heat are that the body does not feel pain, the limbs are not functioning well, the mind is confused but not serious, the voice is weak but comprehensible, and the disease is treatable to this extent. When the condition worsens to the point where he cannot speak, there is no cure.” The clinical characteristics of patients with limb dysfunction in stroke flaccid stage have been clearly described. Modern Chinese medicine practitioners generally believe that the occurrence of limb dysfunction during stroke flaccid paralysis is due to brain damage in patients after stroke, leaving the gods without support and limb loss of regulation.

The etiology and pathogenesis of stroke have been discussed a lot by physicians in the past dynasties, which can be roughly divided into two stages. Most of the physicians before the Tang and Song dynasties supported the view of “external wind.” In his related treatises, Zhang Zhongjing proposed that the cause of the disease is “empty collaterals, wind evils take advantage of the deficiency to enter the middle,” “thieves and evils do not leak, either left or right, righteous qi attracts evil, and deviance fails.” At the same time, the different syndrome differentiation methods of Fengxie in the collaterals, in the meridians, in the fu-organs, and in the viscera have been expounded. After the Tang and Song dynasties, “internal wind” was often used to argue that the sequelae of stroke were mostly virtual and real. Due to the imbalance of qi and blood in the later stage of stroke, the compensation of blood vessels caused hemiplegia, skewed mouth and eyes, etc.

## 4. Experiment of Traditional Chinese Medicine Acupuncture and Moxibustion in the Treatment of Poststroke Limb Dysfunction

### 4.1. Content and Method

#### 4.1.1. Content

From November 2020 to November 2021, patients with upper extremity dysfunction due to phlegm and blood stasis obstruction in the acupuncture clinic and ward of a hospital were selected. Subjects signed informed consent before the experiment. A randomized controlled study design was used, and the Jane's Fugl-Meyer upper extremity motor function score (FMA), the clinical neurological deficit score (NIHSS), the daily living ability score (modified Barthel index), and the upper extremity pain assessment using the visual analog scale (VAS) were used as evaluation indicators before and after treatment. The subjects were treated for a period of 3 months to explore the therapeutic effect of acupuncture combined with pricking and cupping method in the treatment of upper extremity dysfunction caused by phlegm and blood stasis blocking collaterals in stroke. This provides a new and effective method for the rehabilitation of patients with upper extremity dysfunction after stroke, providing evidence-based medicine.

#### 4.1.2. Method

1. Method overview

A total of 83 patients with upper extremity dysfunction due to phlegm and blood stasis blocking collaterals were screened and randomly divided into two groups. The treatment was 5 times a week. One month was a course of treatment, and a total of 3 courses of treatment were observed.

(2) Random method

Eligible cases were determined according to the inclusion criteria and randomly assigned to two groups, using SPSS22.0 statistical analysis system. A simple random number table method was used to make a random allocation card and seal the envelope.

(3) Basic treatment

The two groups of related symptomatic and supportive treatments such as nutritional nerve, energy support, anticoagulation and defibrillation, and blood pressure were the same.

(4) Routine acupuncture treatment in the control group

### 4.2. General Information

A sum of 83 patients were gathered in this preliminary and haphazardly partitioned into 2 groups, 42 in the trial group and 41 in the control group. Among them, 1 patient in the experimental group voluntarily withdrew from the experiment due to intolerance of bleeding, and 1 patient voluntarily withdrew from the experiment due to fear of painful stimulation, and a total of 2 patients dropped out. One person in the control group voluntarily withdrew from the experiment, and a total of one case dropped out. The clinical observation showed that there were 18 males and 22 females in the experimental group and 19 males and 21 females in the control group. The average age of the experimental group was 56.41 ± 6.21 years, and the average age of the control group was 56.20 ± 7.24 years. The disease duration in the experimental group was 6.43 ± 3.06 months, and the disease duration in the control group was 5.88 ± 2.92 months. The number of upper limb pain cases in the experimental group was 11, and the number of upper limb pain cases in the control group was 10. The age of the patients and the course of disease were analyzed by independent samples *t* test. Gender and the number of upper limb pain cases were analyzed by chi-square. After statistical comparison, the difference was not statistically significant (*P* > 0.05), and the two groups had the same baseline and were comparable, as shown in Table 2.

A comparison of clinical study results is shown in Figure 6. From Figure 6, it can be seen that the pain index of the upper limb pain patients in the two groups has obvious changes before and after treatment, and the number of people with a higher general index shows a downward trend.

Table 3 shows that all have improved compared with before treatment, with significant statistical difference (*P* < 0.05). It can be seen that acupuncture and moxibustion have certain curative effects in promoting the recovery of motor function. This indicates that acupuncture and moxibustion have a good promoting effect on improving the motor function of the upper limbs of patients with hemiplegia. Therefore, the use of acupuncture treatment can reduce muscle tension, prevent muscle atrophy, and improve the function of the upper limb on the affected side.

Table 4 shows that all have improved compared with before treatment, with significant statistical difference (*P* < 0.05). It can be seen that acupuncture and moxibustion have good curative effect in promoting the recovery of nerve function. Therefore, acupuncture and moxibustion can relieve blood stasis and phlegm, remove blood stasis, and regenerate. The 3 months after stroke is an important period for neurological recovery. In this case, by using periodic repeated stimulation to establish the corresponding reflex arc, the motor ability of the affected limb is improved, which can help the recovery of the functional nerve defect of the affected side of the upper limb in patients with phlegm and blood stasis blocking collaterals.

### 4.3. Comparison of Curative Effects

Figure 7 shows that after 3 months of treatment, compared with before treatment, there is a significant statistical difference (*P* < 0.05). It shows that acupuncture treatment can promote the improvement of daily living ability of patients. At the same time, the comparison between the groups found that the treatment effect of the experimental group was better than that of the control group, which indicated that after the motor function was improved, the daily living ability of the patients was also improved.

In the experimental group of 40 people, during the treatment of collateral pricking and cupping, 1 case had dizziness, and the patient was instructed to lie down and rest and relieved, and 2 cases of subcutaneous blood stasis were instructed to keep the skin of the treatment area dry and relieved after 1 day.  Figure 8 shows that the VAS scores of the upper appendages on the impacted side of the two groups of patients were lower than those before treatment, and there was a measurably huge distinction (*P* < 0.05). It shows that needle therapy and moxibustion have a decent impact in lessening the aggravation of the upper appendage of the patient. By reducing the release of substance *P*, acupuncture therapy improves the local blood circulation of the upper limb on the affected side and produces a benign response to the structure of joints, muscles, ligaments, and nerves and blood vessels, thereby relieving pain. The results of this study show that acupuncture and moxibustion have a good effect on reducing pain in the upper limbs of patients with hemiplegia.

## 5. Conclusion

The unique two-way regulating effect of acupuncture therapy can not only increase the muscle tension of the limbs of the patients with paralysis but also reduce the muscle tension of the limbs of the patients with paralysis. However, at present, many doctors have expressed their views that the prescription and acupoint selection techniques of acupuncture are very different, and there is no unified standard for acupoint selection. In addition, in the clinical application of acupuncture and moxibustion in the treatment of poststroke limb dysfunction, many physicians ignore the different pathogenesis of stroke in different pathological stages, and always use a set of treatment plans without timely adjustment. In the future, acupuncture treatment of stroke limb function should be more in-depth in terms of syndrome differentiation, prescription selection, acupoint massage, etc., to make it more standardized. Combined with the Bronstrom staging theory, acupuncture can be used to treat poststroke limb dysfunction. From the experimental results, it can be seen that acupuncture combined with collateral pricking and cupping and acupuncture alone have certain curative effects in treating upper extremity dysfunction after stroke. Acupuncture combined with collateral puncturing and cupping alone has a more significant curative effect on upper limb dysfunction after stroke.

## Figures and Tables

**Figure 1:** General model of multivariate influence fusion.

**Figure 2:** Hierarchical structure of image fusion.

**Figure 3:** Pixel-level fusion system architecture.

**Figure 4:** Feature-level fusion system architecture.

**Figure 5:** Architecture of decision-level converged system.

**Figure 6:** Comparison of pain index before and after treatment in two groups of patients with upper limb pain.

**Figure 7:** Comparison of daily living ability scores between the two groups before and after treatment.

**Figure 8:** Comparison of clinical efficacy between the two groups of patients.

**Table 1:** Subjective evaluation criteria.

Fraction	Quality scale	Obstruction scale
5 points	Very nice	No crumbling of picture quality should be visible
4 points	Good	It tends to be seen that the picture quality is weakened; however, it does not impede seeing
3 points	Commonly	It is plainly seen that the picture quality is crumbled and somewhat thwarts seeing
2 points	Difference	Obstruct viewing
1 point	Very poor	Very serious hindrance to viewing

**Table 2:** Comparison of clinical data of two groups of patients.

Group	Number of cases	Age	Course of disease	Gender		Number of upper limb pain cases
				Male	Female	
Test group	40	56.41 ± 6.21	6.43 ± 3.06	18	22	11
Control group	40	56.20 ± 7.24	5.88 ± 2.92	19	21	10
$\frac{t}{x^{2}}$		0.070	0.661	0.058		0.066
*P*		0.944	0.512	0.814		0.796

**Table 3:** Comparison of upper limb FMA scores before and after treatment between the two groups.

	Number of cases	Before treatment ($\bar{X}\pm S$)	After treatment ($\bar{X}\pm S$)
Test group	40	25.41 ± 7.30	34.59 ± 7.62
Control group	40	28.22 ± 5.36	31.33 ± 6.26
*t*		-1.87	2.12
*P*		0.066	0.001

**Table 4:** Comparison of NIHSS scores between the two groups before and after treatment.

	Number of cases	Before treatment ($\bar{X}\pm S$)	After treatment ($\bar{X}\pm S$)
Test group	40	22.31 ± 10.56	13.05 ± 4.30
Control group	40	21.88 ± 9.30	16.62 ± 2.08
*t*		0.18	-3.62
*P*		0.871	0.001

## Data Availability

The datasets generated during and/or analyzed during the current study are not publicly available due to sensitivity and data use agreement.
